RETRACTED

# Mitochondrial ROS Produced by Skeletal Muscle Mitochondria Promote the Decisive Signal for UPRmt Activation

**DOI:** 10.1155/2022/7436577

**Published:** 2022-02-21

**Authors:** Zhe Wang, Hai Bo, Yu Song, Can Li, Yong Zhang

**Affiliations:** ^1^Tianjin University of Sport, Tianjin Key Laboratory of Exercise, Physiology and Sports Medicine, Research Center for Exercise & Health Science, Tianjin 301617, China; ^2^Department of Military Training Medicines, Logistics University of Chinese People's Armed Police Force, Tianjin 300162, China

## Abstract

The **m**itochondrial unfolded protein response (UPRmt) can repair and remove misfolded or unfolded proteins in mitochondria and enhance mitochondrial protein homeostasis. Reactive oxygen species (ROS) produced by regular exercise is a crucial signal for promoting health, and skeletal muscle mitochondria are the primary source of ROS during exercise. To verify whether UPRmt is related to ROS produced by mitochondria in skeletal muscle during regular exercise, we adapted MitoTEMPO, mitochondrially targeted antioxidants, and ROS production by mitochondria. Our results showed that **m**itochondrial ROS is the key factor for activating UPRmt in different pathways.

## 1. Introduction

Regular exercise and physical activity improve physiological ability and body functions [1] and reduce the risk of chronic diseases, including type II diabetes, cardiovascular disease, and cancers [2, 3]. Skeletal muscle is an important part involved in physical activity. Exercise can significantly increase the metabolism of skeletal muscles [4, 5], while contraction of skeletal muscles can produce reactive oxygen species (ROS) [6]. Previous studies have shown that intense exercise and muscle contraction increase ROS production. The damage and modification of cell proteins, lipids, and DNA can lead to skeletal muscle fatigue and injury [7–13]. Therefore, antioxidant supplements are often used as prescriptions to resist the adverse reactions of exercise [14–17]. However, there are increasing evidence to show that exogenous antioxidant supplements have adverse reactions to some acute and chronic responses of skeletal muscles to exercise [18–26], as well as weaken the normal redox signaling pathway in muscles [13], weakening the adaptive response to endurance training [19–21].

Mitochondria are critical for maintaining cell homeostasis by regulating energy production, cell signaling, and apoptosis [27]. Mitochondria are one of the primary sources of ROS during skeletal muscle contraction [28–30]. The mitochondrial unfolded protein response (UPRmt) is a stress response pathway that allows mitochondria to converse with the nucleus, activates the expression of nuclear transcription factors, activates mitochondrial chaperone and proteasome, and promotes the repairing and clearance of misfolded and unfolded proteins, thereby maintaining mitochondrial protein homeostasis and reducing stress response [31–33]. Previous studies have shown that UPRmt in the mitochondrial matrix mainly relies on activating the mitochondrial chaperone HSP60 and the protease CLPP [32, 34–36]. In contrast, UPRmt in the mitochondrial intercellular space (IMS) is associated with the expression of membrane interstitial protein HTRA2 [37–39]. In addition, the antioxidant effect of the UPRmt sirtuin axis is also crucial for the stability of mitochondrial reconstruction protein [35]. To date, there is no report about eliminating the effect of mitochondrial ROS on UPRmt in skeletal muscle mitochondria after long-term exercise. Therefore, we mainly discuss the relationship between the exercise health effect of screening mitochondrial ROS and UPRmt.

RETRACTED

MitoTEMPO is a novel cell-penetrating antioxidant targeting mitochondria, containing a hydrophobic tetramethylpiperidine (TEMPO) group and a lipophilic triphenylphosphine cation (TPP+). It can penetrate mitochondria and remove ROS produced by mitochondria [40–43]. Therefore, we selected MitoTEMPO as a targeted scavenger of mitochondrial ROS and C57BL/6J mice who had long-term exercise and MitoTEMPO were selected as the research objects to explore the effects of skeletal muscle mitochondrial health in mice to investigate the relationship between mitochondrial health and UPRmt and mitochondrial ROS in long-term regular exercise of skeletal muscle MitoTEMPO. Our results showed that during regular exercise, MitoTEMPO offset mitochondrial ROS production by exercise, as the mitochondrial membrane potential of skeletal muscle of mice decreased significantly, and the activation degree of UPRmt mediated by different pathways fell heavily. Therefore, we determined that mitochondrial ROS produced by exercise is one of the important stressors for promoting skeletal muscle health and moderately activated UPRmt is one of the reasons for achieving this health-promoting effect.

## 2. Materials and Methods

### 2.1. Animals

Thirty male C57BL/6J mice (8 weeks old) were purchased from Beijing Vital River Laboratory Animal Technology Co. Ltd. and placed in an environmentally controlled room for a 12-hour light/dark cycle. Prior to the experiment, all animals were given a week of adaptive feeding, which meant that they drink cold and eat without any limitations. All experimental protocols were carried out in accordance with the National Research Council's standards for the care and use of laboratory animals, which had been approved by the Animal Ethics Committee of the Tianjin Institute of Physical Education.

RETRACTED

### 2.2. Exercise Program and MitoTEMPO Intervention

The animals were randomly divided into three groups: control group, exercise group, and exercise + MitoTEMPO group. The exercise group received 2 days of adaptive treadmill training in advance and then 15 m/min treadmill training for 12 consecutive days. MitoTEMPO (Sigma, SML0737) dissolved in normal saline was intraperitoneally injected 0.7 mg/kg into mice to establish the model of the exercise + MitoTEMPO group [44–49]. The rest and exercise groups were injected with the same amount of normal saline as the control group.

### 2.3. Detection of Mitochondrial Membrane Potential

The mice were sacrificed with a broken neck and separate skeletal muscle. Then, they were placed in precooled medium A (120 mM KCL, 5 mM MgCl2.6H2O, 20 mM HEPES, 1 mM EGTA, 0.5% BSA, and pH 7.4). Mince the tissue into small pieces using a pair of sharp scissors (tissue should become a mash), adding medium drops while cutting. Then, the shredded tissue was transferred to a precooled glass homogenizer for grinding and centrifuged at 600 g at 4°C for 10 minutes. The supernatant was transferred to a new centrifuge tube. Next, it was centrifuged at 12000 g at 4°C for 10 minutes, the supernatant was discarded, and mitochondria were resuspended in a small volume of the isolation medium B (300 mM sucrose, 20 mM HEPES,0.1 mM EGTA, and pH 7.4). Then, mitochondria were stored on ice and used within 3–4 h.

After the mitochondria were purified by differential centrifugation, the JC-1 mitochondrial membrane potential detection kit (Beyotime, C2006) was used to detect the mitochondrial membrane potential. When the JC-1 monomer was detected, the excitation light was set at 490 nm and the emission light was set at 530 nm. For detecting JC-1 polymer, the excitation light can be set at 525 nm and the emission light can be set at 590 nm. The larger the JC-1 polymer/monomer ratio, the higher the mitochondrial membrane potential. All the experiments were triplicated.

### 2.4. Western Blotting

RIPA lysis buffer (Beyotime, P0013B) was used to extract total protein from skeletal muscle of mice, and the mixture of the protease and phosphatase inhibitors (Beyotime, P1050) was added. The BCA protein concentration assay kit (Beyotime, P0012) was used to determine the protein concentration. The same number of protein samples was separated using 10% SDS-PAGE electrophoresis and transferred to 0.22 *μ*m PVDF (Millipore, Billerica). Under the condition of room temperature, the PVDF membrane was blocked with 5% skim milk for 1 hour. GDDPH (1 : 1000, Abcam) and *β*-tubulin (1 : 1000, Abcam) were used as internal references, and c-JUN (1 : 800, Abcam), CHOP (1 : 1000, Abcam), HSP60 (1 : 2000, Abcam), CLPP (1 : 2000, Abcam), AKT (1 : 1500, Abcam), pAKT (1 : 1000, Abcam), SIRT3 (1 : 1000, Abcam), and MnSOD (1 : 2000, Abcam) were used as target proteins. The PVDF membrane sealed with milk was incubated with the primary antibody at 4°C overnight, followed by incubation with horseradish peroxidase-labeled secondary antibody at room temperature for 1 hour. After adding Immobilon Western Chemiluminescent HRP Substrate (WBKLS0500, Millipore) in the dark chamber, the protein expression level was recorded by film and the protein grey value was analyzed using ImageJ software. The results were represented by the ratio of the target to an internal reference.

RETRACTED

### 2.5. Statistical Analysis

For statistical analysis, SPSS 23.0 software was used. Variables were tested for normal distribution using the Kolmogorov-Smirnov test. After the test, all the experimental results were in line with the normal distribution and two-way ANOVA was used to test the interaction. The independent sample *t*-test was used for statistical analysis between groups if there was no main effect. Significance was set at a *P* value of less than 0.05 for all experiments.

## 3. Results

### 3.1. Offsetting Mitochondrial ROS Induced in the Loss of Membrane Potential in the Mitochondria of the Training Mice Skeletal Muscle

The mitochondrial membrane potential was measured using the fluorescence labeling method. Compared with the quiet group, 12-day regular exercise increased the mitochondrial membrane potential by 22% (*P* < 0.01), while the mitochondrial membrane potential in skeletal muscle decreased by 17% (*P* < 0.01) after sending MitoTEMPO to eliminate mtROS (Figure 1 and Table 1).

### 3.2. mtROS Is the Key Signal to Activate Mitochondrial Matrix CHOP-Dependent UPRmt

After processing muscle protein, we used Western blot and found that 12-day regular exercise promoted the activation of mitochondrial matrix UPRmt in mice. Our results showed that the mitochondrial chaperone HSP60 and the protease CLPP increased the expression of proteins by 35% (*P* < 0.05) and 13% (*P* > 0.05), respectively. The expression of c-Jun increased by 50% (*P* < 0.01). However, when regular exercise was accompanied by MitoTEMPO intervention, compared with the exercise group, the expression of the above proteins decreased by 35% (*P* < 0.05), 49% (*P* < 0.01), 75% (*P* < 0.01), and 50% (*P* < 0.01) (Figure 2 and Table 2).

### 3.3. mtROS Promoted the Expression of HTRA2 in the Intermembrane Space of Mitochondria

In addition, we found that the expression of AKT and AKT phosphorylation (pAKT) was increased by 70% (*P* < 0.05) and 120%, respectively (*P* < 0.01). In the muscle tissue of mice that regularly exercised for 12 days, the expression of UPRmt-related HTRA2 protein in the mitochondrial membrane cavity was increased by 9% (*P* > 0.05). However, when MitoTEMPO intervention was given during regular exercise, the protein expression of AKT, pAKT, pAKT/AKT, and HTRA2 was decreased by 73% (*P* < 0.05), 119% (*P* < 0.01), 50% (*P* < 0.05), and 43% (*P* < 0.05), respectively (Figure 3 and Table 3).

RETRACTED

### 3.4. mtROS Activated the Expression of MnSOD in the SIRT3-Dominated Antioxidant System

In addition, we also found that the expression of SIRT3 protein in skeletal muscle did not increase significantly after 12 weeks of regular exercise. However, the expression of MnSOD protein in the mitochondrial matrix increased by 67% (*P* < 0.01). Similarly, the expression of SIRT3 and MnSOD in skeletal muscle decreased by 65% (*P* < 0.01) and 62% (*P* < 0.01), respectively, after MitoTEMPO intervention (Figure 4 and Table 4).

## 4. Discussion

Mitochondrial membrane potential is often used as an indicator of mitochondrial membrane integrity to evaluate the health status of mitochondria. Our results show that regular exercise training can improve mitochondrial membrane potential, while MitoTEMPO can significantly reduce the mitochondrial membrane potential after the targeted elimination of mtROS. Thus, the results suggest that mtROS is critical for maintaining mitochondrial membrane potential but how mtROS plays a role in maintaining mitochondrial quality is unclear. UPRmt, as an essential quality control mechanism for maintaining mitochondrial protein homeostasis, is closely related to mitochondrial membrane potential [50–52]. However, whether mtROS generated during exercise is an important signal for UPRmt activation remains to be investigated.

Mitochondria have their chaperone and protease library. When the accumulation of misfolded and unfolded proteins exceeds the folding ability of mitochondria, it can cause damage and organelle dysfunction [53]. Therefore, moderate UPRmt is beneficial to maintain mitochondrial health. Currently, the universal mitochondrial UPRmt reaction occurs in the mitochondrial matrix [54]. The UPRmt reaction mainly depends on the retrograde signal transduction activated by CHOP, leading to the transient expression of nuclear-encoded mitochondrial chaperone HSP60 and the protease CLPP [55], playing a role in controlling protein quality. The degree of this reaction is closely related to the level of unfolded protein in mitochondria [33]. When unfolded or misfolded proteins accumulate in the mitochondrial matrix to produce stress, they are first cleaved by CLPP protease and the peptides are transported out of the mitochondria through an unclear transport mechanism, resulting in the activation of c-Jun N-terminal kinase (JNK2). It stimulates the transcription factor CHOP, and the dimer of CHOP and C/EBP*β* binds to the CHOP element on the promoter of the UPRmt gene, encoding the mitochondrial chaperone protein HSP60 and the protease CLPP [54, 56, 57]. The nucleoencoded mitochondrial chaperone HSP60 mainly helps the further folding of mitochondrial unfolded proteins [58], while the protease CLPP is mainly responsible for the degradation of abnormal proteins in the mitochondrial matrix [55]. In addition, there is a CHOP-independent unfolded protein response UPRmt sirtuin axis in the cytoplasmic matrix and cells can activate the UPRmt sirtuin axis to promote the expression of MnSOD in the matrix and then maintain mitochondrial protein homeostasis [59, 60]. This includes SIRT3, which is located in the mitochondria and controls mitochondrial metabolism [61]. IRT3 regulates the deacetylation of transcription factor FOXO3A, which causes FOXO3A to localize in the nucleus [62–64], stimulating the transcription of mitochondrial superoxide dismutase 2 (MnSOD) [65, 66], and then has an antioxidant role. A previous study has shown that CHOP gene knockout and SIRT3 inhibition mediated by RNAi do not affect the classical UPRmt transcription reaction [51]. Therefore, the UPRmt reaction involved in the SIRT3-FOXO3A axis is independent of the mitochondrial quality control system of CHOP and the antioxidant activity of the UPRmt sirtuin axis may be highly complementary to the classical UPRmt transcription reaction to ensure mitochondrial health [52]. Our results showed that exercise activated the mitochondrial matrix UPRmt response and increased the content of MnSOD. However, the expression of c-JUN,CHOP, HSP60,CLPP, SIRT3, and MnSOD decreased differently after applying MitoTEMPO to inhibit mtROS, suggesting that our mtROS is a key factor for exercise to promote CHOP-dependent and as sirtuin axis-based UPRmt.

RETRACTED

Unfolded protein protection programs are also present in the mitochondrial intermembrane compartment (IMS) [54]; IMS protein quality control is different from matrix protein protection procedures. The control is divided into two sections. First, misfolded proteins targeting IMS are ubiquitinated and degraded by the 26S proteasome in the cytoplasm. Second, when unfolded proteins and excessive proteins enter IMS, they can be eliminated by the protease HTRA2 (also known as OMI) [67]. The specific process is that the phosphorylation of protein kinase B (AKT) can be activated when there is an excessive accumulation of misfolded or unfolded proteins in the mitochondrial membrane intercellular space (IMS); thus, estrogen receptor *α* (ER*α*) in the nucleus is activated and the expression of IMS protease HTRA2 is induced to control the quality of IMS protein [68]. Our results show that exercise activates the mitochondrial matrix UPRmt-related protein HTRA2 by upregulating AKT and pAKT, while the expression of AKT, pAKT, and HTRA2 is suppressed after blocking out mtROS, suggesting that exercise-generated mtROS is an important signal for activating IMS UPRmt.

## 5. Conclusion

Regular exercise training generates mtROS as a key signal to activate different pathway-dependent UPRmt. The production of appropriate amounts of mtROS enhances protein homeostasis in mitochondria which can maintain the integrity of mitochondrial membranes and safeguard the efficiency of energy metabolism.

## Figures and Tables

**Scheme 1:** MitoTEMPO molecular formula: C29H35N2O2P · Cl [H2O].

**Figure 1:** JC-1 polymer/monomer ratio. Reflect changes in mitochondrial membrane potential. After regular exercise, mitochondrial membrane potential increased but this phenomenon disappeared after the application of MitoTEMPO. Control, *n* = 8; exercise, *n* = 8; exercise treated with MitoTEMPO, *n* = 8. ∗∗*P* < 0.01.

**Figure 2:** Chop-dependent UPRmt-related protein expression in the mitochondrial matrix. Control, *n* = 8; exercise, *n* = 8; exercise treated with MitoTEMPO, *n* = 8. ^∗^*P* < 0.05 and ^∗∗^*P* < 0.01.

**Figure 3:** UPRmt-related protein expression in the intermembrane space of mitochondria. Control, *n* = 8; exercise, *n* = 8; exercise treated with MitoTEMPO, *n* = 8.∗*P* < 0.05 and ^**^P < 0.01.

**Figure 4:** Changes of the UPRmt sirtuin axis-related protein expression. Control, *n* = 8; exercise, *n* = 8; exercise treated with MitoTEMPO, *n* = 8. ^∗^*P* < 0.05 and ^∗∗^*P* < 0.01.

**Table 1:** Comparison of mitochondrial membrane potential among three groups ($\overset{-}{X}\pm \text{SD}$).

Group	JC-1 polymer	JC-1 monomer	JC-1 polymer/monomer ratio
Control	43736 ± 4354.87	51618.5 ± 4891.14	0.847 ± 0.029
Exercise	43623.75 ± 1830.03	41086.75 ± 1634.99	1.062 ± 0.03^∗∗^
Exercise + MitoTEMPO	42852.75 ± 3422.52	48085.25 ± 5935.12	0.895 ± 0.048^##^

^∗∗^ *P* < 0.01 vs control; ^##^*P* < 0.01 vs exercise.

**Table 2:** Mitochondrial matrix CHOP-dependent UPRmt protein and control group normalization ($\overset{-}{X}\pm \text{SD}$) results.

Relative expression of protein	Control	Exercise	Exercise + MitoTEMPO
c-JUN	1 ± 0.298	1.506 ± 0.161^∗∗^	1.15 ± 0.16^#^
CHOP	1 ± 0.102	1.076 ± 0.068	0.589 ± 0.17^##^
HSP60	1 ± 0.219	1.347 ± 0.174^∗^	0.603 ± 0.136^##^
CLPP	1 ± 0.102	1.129 ± 0.067	0.624 ± 0.168^##^

^∗^ *P* < 0.05 and ^∗∗^*P* < 0.01 vs control and ^#^*P* < 0.05 and ^##^*P* < 0.01 vs exercise.

RETRACTED

**Table 3:** HTRA2 in the intermembrane space of mitochondria protein and control group normalization ($\overset{-}{X}\pm \text{SD}$).

Relative expression of protein	Control	Exercise	Exercise + MitoTEMPO
AKT	1 ± 0.305	1.722 ± 0.229^∗^	0.991 ± 0.430^#^
pAKT	1 ± 0.361	2.228 ± 0.255^∗∗^	1.034 ± 0.11^##^
pAKT/AKT	1 ± 0.154	1.394 ± 0.329	0.782 ± 0.193^#^
HTRA2	1 ± 0.145	1.092 ± 0.06	0.661 ± 0.205^#^

^∗^ *P* < 0.05 and ^∗∗^*P* < 0.01 vs control and ^#^*P* < 0.05 and ^##^*P* < 0.01 vs exercise.

**Table 4:** MnSOD in SIRT3 dominated antioxidant system protein and control group normalization ($\overset{-}{X}\pm \text{SD}$).

Relative expression of protein	Control	Exercise	Exercise + MitoTEMPO
SIRT3	1 ± 0.119	0.98 ± 0.157	0.324 ± 0.036^##^
MnSOD	1 ± 0.155	1.668 ± 0.125^∗∗^	1.051 ± 0.157^##^

^∗∗^ *P* < 0.01 vs control and ^##^*P* < 0.01 vs exercise.

## Data Availability

The datasets used and/or analyzed during the current study are available from the corresponding author upon reasonable request.
